The article "Protective and antidiabetic effects of extract from Nigella sativa on blood glucose concentrations against streptozotocin (STZ)-induced diabetic in rats: an experimental study with histopathological evaluation" was retracted in 2016. Reasons: misconduct by an author; plagiarized text; compromised peer review; false authorship.

# Protective and antidiabetic effects of extract from *Nigella sativa* on blood glucose concentrations against streptozotocin (STZ)-induced diabetic in rats: an experimental study with histopathological evaluation

**DOI:** 10.1186/1746-1596-8-137

**Published:** 2013-08-15

**Authors:** Samad Alimohammadi, Rahim Hobbenaghi, Javad Javanbakht, Danial Kheradmand, Reza Mortezaee, Maryam Tavakoli, Farshid Khadivar, Hamid Akbari

**Affiliations:** 1 Department of Physiology, Faculty of Veterinary Medicine, Tehran University, Tehran, Iran; 2 Department of Pathology, Faculty of Veterinary Medicine, Urmia University, Urmia, Iran; 3 Department of Pathology, Faculty of Veterinary Medicine, Tehran University, Tehran, Iran; 4 Faculty of Medicine MD, Graduate Student of Islamic Azad University of Mashhad, Mashhad, Iran; 5 Young Researchers Club and Elites, Mashhad Branch, Islamic Azad University, Mashahd, Iran; 6 Graduate Faculty of Veterinary Medicine, Urmia University, Urmia, Iran; 7 Faculty of Veterinary Medicine, Tehran University, Tehran, Iran; 8 Department of Clinical Science, Faculty of Veterinary Medicine, Urmia University, Urmia, Iran

**Keywords:** *Nigella Sativa*, Streptozotocin, Hypoglycemic, Rat

## Abstract

**Background:**

Diabetes in humans induces chronic complications such as cardiovascular damage, cataracts and retinopathy, nephropathy and polyneuropathy. The most common animal model of human diabetes is streptozotocin (STZ)-induced diabetes in the rat. The present study investigated the effects of *Nigella sativa* hydroalcholic extract on glucose concentrations in streptozotocin (STZ) diabetic rats.

**Methods:**

In this study Twenty-five Wister-Albino rats (aged 8-9 weeks and weighing 200-250 g) were tested. Rats were divided into five experimental groups (control, untreated STZ-diabetic (60 mg/kg B.W., IP), treated STZ-diabetic with hydroalcholic extract of *Nigella Sativa* (NS) (5 mg/kg B.W, IP), treated STZ-diabetic with hydroalcholic extract of NS (10 mg/kg B.W., IP) and treated STZ-diabetic with hydroalcholic extract of NS (20 mg/kg B.W., IP and 32 days were evaluated to assess its effect on fasting blood glucose (FBG), and in different groups fasting blood glucose (FBG) and body weight (BW) were measured in the particular days (1, 16 and 32). At the end of the study, the animals were fasted overnight, anaesthetized with an intraperitoneal injection of sodium pentobarbital (60 mg/kg), and sacrificed for obtaining tissues samples (liver, pancreases). The number of islets and cells were counted and the islet diameters were determined by calibrated micrometer. The glycogen content in the liver was examined by Periodic Acid-Schiff (PAS) staining.

The article "Protective and antidiabetic effects of extract from Nigella sativa on blood glucose concentrations against streptozotocin (STZ)-induced diabetic in rats: an experimental study with histopathological evaluation" was retracted in 2016. Reasons: misconduct by an author; plagiarized text; compromised peer review; false authorship.

**Results:**

Treatment with NS (5 mg/kg b.w.) markedly increased BW gain and the FBG level was significantly (p<0.001) reduced when compared to the control. Histopathological examination showed that the NS (5 mg/kg b.w.) partially recovered hepatic glycogen content and protected the great deal of the pancreatic islet cells. The number of islets, cells and islets diameter were found statistically significant when compared to the control (p<0.01, p<0.05).

**Conclusions:**

Higher doses of NS did not exhibit any therapeutic effect. These results showed that hydroalcholic extract of NS at low doses has hypoglycemic effect and ameliorative effect on regeneration of pancreatic islets and may be used as a therapeutic agent in the management of diabetes mellitus. The hypoglycemic effect observed could be due to amelioration of β-cell, thus leading to increased insulin levels. Consequently, *N. sativa* may prove clinically useful in the treatment of diabetics and in the protection of β-cells against streptozotocin.

**Virtual slide:**

The virtual slide(s) for this article can be found here: http://www.diagnosticpathology.diagnomx.eu/vs/1845133011104231

## Background

*Nigella sativa L.*, commonly known as black seed, belongs to the botanical family Ranunculaceae. It has being used in countries bordering the Mediterranean Sea, Pakistan, India and Iran, as a natural remedy for over 2000 years [1]. Black seed components display a remarkable array of biochemical, immunological and pharmacological actions, including bronchodilatory [2], anti-inflammatory [3], antibacterial [4], hypoglycaemic [5] and immunopotentiating effects [6].

*N. sativa* extract has been shown to possess immunopotentiating, anti-oxidant, anti-tumoral, and anti-diabetic properties. The oil of *N. sativa* exhibits analgesic and anti-inflammatory effects in rats. Most of these properties have been attributed mainly to the quinone constituents of *N. sativa*, of which thymoquinone is the main active ingredient of the volatile oil isolated from the black seeds. Thymoquinone has been shown to possess strong antioxidant properties and to suppress the expression of inducible NO synthase in rat macrophages [7].

Many studies have also examined the anti-diabetic effect of *N. sativa* in diabetic animal models. Aside from the effect of its crude aqueous extract to restore glucose homeostasis. *N. sativa* petroleum ether extract significantly lowered fasting plasma levels of insulin and triglycerides and normalized HDL-cholesterol. In this latter study by Le and collaborators, *N. sativa* was also shown to enhance liver cell insulin sensitivity [1,3,7].

β cell defect and insulin resistance are essential features of non-insulin-dependent diabetes mellitus (NIDDM) and both features are the focus of intensive investigations. In this context, plants are source of many biochemical substances that present interesting therapeutic properties. Some plants with anti-diabetic properties have been in use in many Middle Eastern countries as a natural remedy for diabetes in traditional medicine; *N. sativa* is one of these plants. It has a great potential in the treatment of diabetic animals because of its combined hypoglycemic [2,4,7].

The article "Protective and antidiabetic effects of extract from Nigella sativa on blood glucose concentrations against streptozotocin (STZ)-induced diabetic in rats: an experimental study with histopathological evaluation" was retracted in 2016. Reasons: misconduct by an author; plagiarized text; compromised peer review; false authorship.

In earlier experiments we have shown that streptozotocin, given at 45 days post-infection (dpi) affected the morphology of the reproductive organs of male and female worms and lowered the number of viable eggs in the intestine and the amount of eggs in the feces. However, the morphological changes were caused directly by the drug [5-7].

STZ, an antibiotic produced by Streptomyces achromogenes, is the most commonly used agent in experimental diabetes. The mechanism by which STZ destroys β-cells of the pancreas and induces hyperglycemia is still unclear. Many actions have been attributed to STZ that are similar to those that have been described for the diabetogenic action of alloxan, including damage to pancreatic β-cell membranes and depletion of intracellular nicotinamide adenine dinucleotide (NAD) in islet cells. In addition, STZ has been shown to induce DNA strand breaks and methylation in pancreatic islet cells [8,9]. Its diabetogenic action has been ascribed to an increase in the intracellular methylation reaction, DNA strand breaks, and the production of nitric oxide (NO) and free radicals.NO is involved in pancreatic destruction, where the interaction between NO and ROS modulates oxidative damage. STZ can be used to induce different types of diabetes. For example, to produce experimental models of Type 1 diabetes, mice are treated with high doses of STZ, which depletesb -cells [8,10,11].

It is known that people suffering from diabetes mellitus are related to higher incidence of bacterial and fungal infections. Diabetes Mellitus is a chronic disease which affects the metabolism of proteins, carbohydrates and lipids. The major characteristic is hyperglycaemia as a consequence of abnormal secretion of insulin in the pancreas (type I) or inefficient action of insulin in the target tissues (type II) [12]. Type 2 diabetes is sharply increasing globally, including in many parts of the developing world, in major part as a consequence of the worldwide “epidemic” of obesity. For centuries, prior to and after the discovery of insulin, medicinal plants have been used to normalize glycemia in diabetic patients. This disorder promotes adverse effects in all organic systems. Diabetes exerts a negative action on the neuroendocrine axis and those effects can enhance the action of diabetes on other organs that are dependent on the axis [12].

The article "Protective and antidiabetic effects of extract from Nigella sativa on blood glucose concentrations against streptozotocin (STZ)-induced diabetic in rats: an experimental study with histopathological evaluation" was retracted in 2016. Reasons: misconduct by an author; plagiarized text; compromised peer review; false authorship.

Diabetics and experimental animal models of diabetes exhibit high oxidative stress due to persistent and chronic hyperglycemia, which may deplete the activity of the anti-oxidative defense system and promote the generation of free radicals [12]. Streptozotocin (STZ) is frequently used to induce diabetes in experimental animals through its toxic effects on pancreatic β -cell [13] and as a potential inducer of oxidative stress. It has been reported that diabetes induced by STZ is the best characterized system of xenobiotic-induced diabetes and the commonly used model for the screening of anti-hyperglycemic activities [14].

The present study was designed to investigate the mechanism(s) of the hypoglycaemic effect of *N. sativa* hydroalcholic extract, especially with respect to hepatic gluconeogenesis, and to investigate its possible streptozotocin effects in diabetic rats.

## Methods

### Experimental procedure

#### Plant material and extraction procedure

The NS seeds were purchased from a local herb store in Urmia, Iran. The specimens have been kept at the Department of Pathology, Veterinary Medicine Faculty, Urmia University, Iran. The seeds of NS were powdered by a grinder. Subsequently, 20 g of the powdered seeds were added to 400 ml of distilled water, and the extraction was obtained by steam distillation. The distillation process was continued until 200 ml of distillate was collected. The distillate was extracted three times with chloroform [15].

#### Chemicals and streptozotocin-induced diabetes

Streptozotocin was purchased from Sigma chemical Co. Other chemicals were purchased from Merck Company (Germany). Diabetes mellitus was induced by single intraperitoneal (IP) injection of freshly prepared STZ at dose of 60 mg/kg b.w. dissolved in 0.01 M citrate buffer, pH 4.5. After 24 h of STZ injection, and overnight fast, blood was taken from tail artery of the rats. Animals with FBG level of higher than 250 mg/dl were selected for the diabetic groups.

#### Animals

In current study, 25 Wister-albino rats of both sexes, weighing 160-200 g with averagely 32 days old were utilized. The animals were kept in individual propylene cages under standard laboratory conditions by the dimensions of 30×50×25 cm^3^ two by two. Rats were maintained on a 12 hour light/dark cycle at 22± 1°C and 50± 10% humidity. The animals were kept in standard room conditions and fed with standard rat diet and water ad libitum. All animals received human care according to the criteria outlined in the “Guide for the Care and Use of Laboratory Animals” prepared by the National Academy of Sciences and published by the National Institutes of Health.

The article "Protective and antidiabetic effects of extract from Nigella sativa on blood glucose concentrations against streptozotocin (STZ)-induced diabetic in rats: an experimental study with histopathological evaluation" was retracted in 2016. Reasons: misconduct by an author; plagiarized text; compromised peer review; false authorship.

#### Experimental design and sample collection

Rats were divided into five groups (n = 5 in each group). Diabetes was induced in all groups except the control group by a single intraperitoneal (i.p.) injection of STZ (60 mg⁄kg) freshly dissolved in 5 mmol⁄L citrate buffer (pH 4.5), as described previously [16]. One day after STZ injection, diabetes was confirmed by measuring blood glucose levels in blood samples from the tail vein with a One Touch Glucometer (Life scan; Johnson & Johnso, New Brunswick, NJ, USA). Rats with blood glucose levels 250 mg ⁄dL were considered diabetic. Detailed descriptions of the five groups are as follows: Group A (control group), rats were injected with an equal volume of vehicle (citrate buffer); Group B, untreated STZ-diabetic (60 mg/kg b.w., IP); Group C, treated STZ-diabetic with hydroalcholic extract of NS (5 mg/kg b.w., IP); Group D, treated STZ-diabetic with hydroalcholic extract of NS (10 mg/kg b.w., IP); Group E, and treated STZ-diabetic with hydroalcholic extract of NS (20 mg/kg b.w., IP), and 32 days were evaluated to assess its effect on fasting blood glucose (FBG), and in different groups fasting blood glucose (FBG)and body weight (BW) were measured in the particular days (1, 16 and 32).

#### Histological examinations

The rats were euthanized by a lethal dose of sodium pentobarbital. The histopathological samples (liver and pancreas) were fixed in 10% neutral buffered formalin. Fixed tissue samples were processed routinely by the paraffin embedding technique. In Histopathology, the number of islets and the number of islet cells of each islet were counted. The islet diameters were measured using calibrated micrometer by taking of fixed number of islets in all groups.

#### Statistical analysis

All data were expressed as mean ± SD. Statistical analysis of data for BW and BG was performed one-way analysis of variance (ANOVA) followed by Tukey’s post hoc test for multiple comparisons was used to compare differences among experimental groups. The statistical analysis of data for the number of islets and the number of islet cells and islets diameter (μm) in pancreatic tissues was done using one-way analysis of variance (SPSS 21.0) followed by Tukey post hoc test. P values of less than 0.05 were considered as significant.

## Results

### Effect of *N. sativa* extract on body weight

Effect of hydroalcholic extract of *N. sativa* on body weight in STZ-induced diabetic rats were summarized in the Table 1. The changes of rat body weights in five groups were investigated. There was a progressive increase in the body weight in the control and a progressive decrease in the STZ group, whereas the body weight in the STZ+ NS groups (3, 4, 5) showed a progressive decrease (Table 1). Administration of NS attenuated the weight loss induced by STZ injection in rats. In the present experimental condition, the treatment of STZ+ NS alone had no significant effect on changes in body weight. The mean BW of animals in group 1, 2 and 3 at the 16th day of this study were 201, 182.4 and 192.2 respectively while at 32th day of the study they were found to be 204.4, 168.8 and 185.2 respectively. (Group 2, 4 and 5; Table 1).

The article "Protective and antidiabetic effects of extract from Nigella sativa on blood glucose concentrations against streptozotocin (STZ)-induced diabetic in rats: an experimental study with histopathological evaluation" was retracted in 2016. Reasons: misconduct by an author; plagiarized text; compromised peer review; false authorship.

**Table 1:** Effect of hydroalcholic extract of *N. sativa* on body weight in STZ-induced diabetic rats

**Groups**	Treatment groups*	**Body weight**		
		**Day 1**	**Day 16**	**Day 32**
1	Control	197.4 ± 4.9	201 ± 5.6 ^c^	204.4 ± 5.7
2	STZ	195.6 ± 6.4	182.4 ± 6.3 ^a^	168.8 ± 7.4 ^a^
3	STZ+ NS 5 mg/kg b.w	198.4 ± 3.6	192.2 ± 3.3 ^b d^	185.2 ± 5.1 ^a c^
4	STZ+ NS 10 mg/kg b.w	197.6 ± 24	185.8 ± 2.8 ^a e^	176.2 ± 3.1 ^a e^
5	STZ+ NS 20 mg/kg b.w	196 ± 3.3	183 ± 22 ^a e^	170.8 ± 1.9 ^a e^

* Values are means ± SD (n5). ^a^ p 0.001 comparison to control; ^b^ p 0.01 comparison to control; ^c^ p 0.001 comparison to STZ; ^d^ p 0.05 comparison to STZ; ^e^ not significant comparison to STZ. The data were analyzed using One-way-ANOVA analysis and Tukey’s post hoc test.

### Effect of *N. sativa* extract on blood glucose

Effect of hydroalcholic extract of *N. sativa* on blood glucose in STZ-induced diabetic rats were summarized in the Table 2. Table 2 shows change in blood glucose levels of control and diabetic rats during the experimental period. After STZ and STZ+ NS injections, the blood glucose levels of 2, 3, 4 and 5 groups significantly increased (P <0.001) and P<0.01). The means ± SD of blood glucose concentrations before of STZ injection and before administration of *N. sativa* (in treatment groups) were 131.4 2.3, 464.2 43.5, 428.8 35.9, 435.4 50.7 and 446.2 41.1 mg/dl in control, STZ and STZ+ NS groups (5, 10, 20 mg/kg b.w), respectively. 16 days after injection of STZ, the mean±SE of blood glucose concentration were 480.6 35.3, 361 36, 475.8 36.2 and 482 28.5 mg/dl in STZ and STZ+ NS (5,10,20 mg/kg b.w) groups, respectively.

**Table 2:** Effect of hydroalcholic extract of *N. sativa* on blood glucose in STZ-induced diabetic rats

**Groups**	Treatment groups*	**Blood glucose**		
		**Day 1**	**Day 16**	**Day 32**
1	Control	131.4 ± 2.3	132.4 ± 3.2	123.6 ± 4.9
2	STZ	464.2 ± 43.5 ^a^	480.6 ± 35.3 ^a^	565.4 ± 30.9 ^a^
3	STZ+ NS 5 mg/kg b.w	428.8 ± 35.9 ^a^	361 ± 36 ^b^	323.2 ± 32.2 ^b^
4	STZ+ NS 10 mg/kg b.w	435.4 ± 50.7 ^a^	475.8 ± 36.2 ^c^	513.2 ± 42.7 ^c^
5	STZ+ NS 20 mg/kg b.w	446.2 ± 41.1 ^a^	482 ± 28.5 ^c^	517.6 ± 27.3 ^c^

* Values are means ± SD (n5). ^a^ p 0.001 comparison to control; ^b^ p 0.01 comparison to STZ; ^c^ not significant comparison to STZ. The data were analyzed using One-way-ANOVA analysis and Tukey’s post hoc test.

The article "Protective and antidiabetic effects of extract from Nigella sativa on blood glucose concentrations against streptozotocin (STZ)-induced diabetic in rats: an experimental study with histopathological evaluation" was retracted in 2016. Reasons: misconduct by an author; plagiarized text; compromised peer review; false authorship.

The effect of STZ in 16 days showed a gradually increasing of blood glucose level which it was (480.6 35.3) in 2 week and it reached to (565.4 30.9) mg/dl during 32 days after injection of STZ. The mean±SE of Blood Glucose concentration level in STZ+ NS) groups (5, 10, 20 mg/kg b.w) decreased from 323.2 32.2, 513.2 42.7 and 517.6 27.3 mg/dl in the 32 days (Table 2). These results suggest that 5 mg/kg b.w. is the most effective dose for assessing the anti-hyperglycemic potential of hydroalcholic extract of NS in diabetic rats. However, higher doses up to 20 mg/kg b.w. did not exhibit any dose dependent effect. Treatment with NS (5 mg/kg b.w.) markedly increased BW gain and the FBG level was significantly (p<0.001) reduced when compared to the control.

### Histopathological findings

Histopathological study of islets of Langerhans revealed that size of Langerhans islets in diabetic control group had a significant difference in comparison with all treatment groups (P < 0.05). There was no significant difference in size of Langerhans islets between the treated rats (with STZ+ NS) and STZ rats.

Effect of hydroalcholic extract of *N. sativa* on the number of islets and the number of islet cells and islets diameter (μm) in pancreatic tissues in rats were summarized in the Table 3. Light microscopy evaluation of the pancreas of control rats (Group 1) showed normal pancreatic islet structure (Figure 1A). In contrast, sections of the pancreas from untreated diabetic rats (Group 2) disclosed that the islets were comparatively small and shrunken and the islet cells were degenerated (hydropic degeneration) and necrotized (Figure 1A) (Table 3). *N. sativa* treatment at dose of 5 mg/kg b.w. (Group 3) protected the great deal of the Langerhans islet cells. Nevertheless, light hydropic degeneration and necrosis were seen in the remaining cells (Figure 1C). *N. sativa* treatment at doses of 10 and 20 mg/kg b.w. did not show significant difference comparison to untreated diabetic rats (Table 3). The histochemical PAS staining demonstrated that STZ-induced diabetes resulted in approximately complete depletion of hepatic glycogen in comparison to the control group (Figure 1A,B). NS treatment at dose of 5 mg/kg b.w (Group 3) partially recovered the hepatic glycogen content (Figure 1C). Treatment with NS extract at doses of 10 and 20 mg/kg b.w. did not show remarkable change in hepatic glycogen content (Figure 1D).

The article "Protective and antidiabetic effects of extract from Nigella sativa on blood glucose concentrations against streptozotocin (STZ)-induced diabetic in rats: an experimental study with histopathological evaluation" was retracted in 2016. Reasons: misconduct by an author; plagiarized text; compromised peer review; false authorship.

**Table 3:** Effect of hydroalcholic extract of *N. sativa* on the number of islets and the number of islet cells and islets diameter (μm) in pancreatic tissues in rats

**Groups**	Treatment groups*	**Islets**	**Cells**	**Islets diameter (μm)**
1	Control	19.2 ± 4.9 ^d^	120.4 ± 24.6 ^d^	102.8 ± 11.8 ^d^
2	STZ	5 ± 1.4 ^a^	42 ± 7.3 ^a^	51.8 ± 16.3 ^a^
3	STZ+ NS 5 mg/kg b.w	13.6 ± 4.5 ^g e^	85.6 ± 19.4 ^c e^	84.4 ± 21.5 ^g f^
4	STZ+ NS 10 mg/kg b.w	6 ± 1.5 ^a h^	47.6 ± 14.1 ^a h^	63.4 ± 13.5 ^b h^
5	STZ+ NS 20 mg/kg b.w	5.4 ± 1.1 ^a h^	49.2 ± 14.1 ^a h^	57.2 ± 12 ^b h^

* Values are means ± SD (n5). ^a^ p 0.001 comparison to control; ^b^ p 0.01 comparison to control; ^c^ p 0.05 comparison to control; ^d^ p 0.001 comparison to STZ; ^e^ p 0.01 comparison to STZ; ^f^ p 0.05 comparison to STZ; ^g^ not significant comparison to control; ^h^ not significant comparison to STZ. The data were analyzed using One-way-ANOVA analysis and Tukey’s post hoc test.

**Figure 1:** **Histopathological study of islets of Langerhans and effect of hydroalcholic extract of *N. sativa *on the number of islets and the number of islet cells and islets diameter (μm) in pancreatic tissues in rats. A**- Diabetic group, shrunken islets of Langerhans displaying degenerative and necrotic changes and vacuolization in diabetic rats without treatment (H&E × 400); **B**- NS treated group (5 mg/kg b.w.). NS protected the majority of cells in the islet of Langerhans. However, the remaining cells exhibit light hydropic degeneration, degranulation, and necrosis. In addition, a few cells with a picnotic nucleus are indicated (H&E × 400). **C**- Complete glycogen depletion is seen due to STZ-induced diabetes (PAS staining × 400) and The hepatic glycogen level remarkably elevated after 32 days treatment with NS at dose of 5 mg/kg b.w. (PAS staining × 400). **D**- The hepatic glycogen content did not change considerably after 32 days treatment with NS at dose of 10 and 20 mg/kg b.w. (PAS staining × 400).

## Discussion

Diabetes mellitus is a chronic, systemic, metabolic disease defined by hyperglycemia and characterized by alterations in the metabolism of carbohydrate, protein and lipid. Oxidative stress thought to be increased in a system where the rate of free radical production is increased and/or the antioxidant mechanisms are impaired. In recent years, the oxidative stress-induced free radicals have been implicated in the pathology of insulin dependent diabetes mellitus [3,5,8-10].

In our study, a significant weight loss was observed in the diabetic group while NS treated (5 mg/kg b.w.) rats exhibited significant increase in the BW in comparison to diabetic group (Group 2) but was lower than in the normal controls. This effect on the BW was not observed at higher doses of extract. This finding is in agreement with Kanter et al., 2004 reported that NS markedly improved BW gain in STZ-induced diabetic rats. A possible explanation for this might be that NS reduces hyperglycemia, and therefore protein wasting due to inaccessibility of carbohydrate does not occur [17].

The article "Protective and antidiabetic effects of extract from Nigella sativa on blood glucose concentrations against streptozotocin (STZ)-induced diabetic in rats: an experimental study with histopathological evaluation" was retracted in 2016. Reasons: misconduct by an author; plagiarized text; compromised peer review; false authorship.

In present study, the hydroalcholic extract of NS at dose of 5 mg/kg b.w. revealed a significant hypoglycemic effect in STZ-induced diabetic rats by diminishing the FBG levels. The FBG lowering effect of that was further increased after 32 day treatment. In addition, results showed that the anti-hyperglycemic effect of the NS extract is time dependent. This finding is in agreement with Fararh et al., 2002 [18].

In present study, the lowering effects of black seed oil on blood glucose were correspondent with the previous trials. Some studies have been conducted on the characterization of the bioactives and mechanisms mediating its anti-hyperglycemic action. In an experimental study, Alsaif [19] reported that blood glucose lowering effect of black seed oil was due to improved insulin insensitivity in diabetic rats. Another study proposed its hypoglycemic effect is due to improved extrapancreatic actions of insulin rather than by stimulated insulin release [20]. Furthermore, Abdelmeguid et al. [21] reported that the anti-hyperglycemic effect of black seed oil and its active component thymoquinone could be due to reduction of oxidative stress, thus preserving pancreatic β -cell integrity lead to insulin levels increase. Furthermore, the black seed oil contains many bioactive constituents such as thymoquinone, p-cymene, pinene, dithymoquinone and thymohydroquinone [22].

The increase in glycogen levels could be due to the antidiabetic activity of NS, streptozotocin induces degeneration of the pancreas with a lobular atrophy and a decline in size and number of Langerhans islets [23,24]. In this study, the damage of pancreas in STZ treated diabetic rats and regeneration of Langerhans islets by NS extract was observed. Furthermore, the number of islets, islet cells and islets diameter significantly increased in NS (5 mg/kg b.w.) treated group compared to STZ-induced diabetic group. However, there have been no morphometric studies to date examining the pancreatic structure in STZ-diabetic rats treated with NS extract. Histopathlogically, treatment with the hydroalcholic extract of NS (5 mg/kg b.w.) revealed partial regeneration of the islet cells with light hydropic degeneration and necrosis in the remaining cells. These findings are in accordance with the results reported by Kanter et al. [17].

The article "Protective and antidiabetic effects of extract from Nigella sativa on blood glucose concentrations against streptozotocin (STZ)-induced diabetic in rats: an experimental study with histopathological evaluation" was retracted in 2016. Reasons: misconduct by an author; plagiarized text; compromised peer review; false authorship.

Measurement of the effect of *N. sativa* on gluconeogenesis and liver glucose production helps to clarify part of the hypoglycemic mechanism since hepatic glucose production through gluconeogenesis is known to contribute to hyperglycemia in diabetic patients. Research on isolated hepatic cells showed a significant decrease in glucose production from gluconeogenic elements like glycerol, alanine and lactate in *Nigella sativa* oil-treated animals as compared to the untreated animals [3-5]. This significant decrease in liver glucose output and ameliorative effect on regeneration of pancreatic islets suggests that the observed antidiabetic action of *N. sativa* is at least partially mediated through an effect on hepatic gluconeogenesis.

## Conclusions

In conclusion, based on the experimental findings, it was suggested that administration of *N. sativa*, at a safe dose level, suppresses STZ-induced diabetic in the rat. We believe that further preclinical research into the utility of *N. sativa* treatment may indicate its usefulness as a potential treatment in diabetic patients, our results suggested that hydroalcholic extract of NS at low doses has beneficial effect on FBG level and ameliorative effect on regeneration of pancreatic islets and may be used as a therapeutic agent in the management of diabetes mellitus.

## Competing interests

The authors declare that they have no competing interests.

## Authors’ contributions

SA and RH participated in the histopathological evaluation, performed the literature review, acquired photomicrographs and drafted the manuscript and gave the final histopathological diagnosis and designed and carried out all the experiments. JJ is the principal investigator of the laboratory in which the research was performed and contributed to the interpretation of the data and writing of the manuscript. DKH, RM, FKH, MT and HA edited the manuscript and made required changes and wrote the manuscript. All authors have read and approved the final manuscript.
